# Automatic Scoring for Translations Based on Language Models

**DOI:** 10.1155/2022/2171206

**Published:** 2022-06-28

**Authors:** Diming Wu, Mingke Wang, Xiaomin Li

**Affiliations:** ^1^School of Foreign Language, Bengbu University, Bengbu, China; ^2^College of Computer Science and Technology/College of Artificial Intelligence, Nanjing University of Aeronautics and Astronautics, Nanjing, China

## Abstract

With the development of English education, translation scoring has gradually become a time-consuming and energy-consuming task, and it is difficult to ensure objectivity because of the subjective factors in manual correcting. Due to the similarity between the quality evaluation of responses generated by the dialogue system and the translation results submitted by students, we selected two metrics of dialogue to automatically score the translations, which are applied in a case study. The experiments show that the hybrid scores of two metrics are close to human scores. In conclusion, the method is feasible to apply the evaluation metrics of dialogue systems to translation scoring, and it can provide an improvement idea for the automatic scoring of translations in the future.

## 1. Introduction

Translation is playing an important part in English education. It is also unavoidable for teachers to score the translation results submitted by students, such as ordinary translation homework and translation questions in examinations. However, teachers have encountered the following problems in the process of scoring the translation answers: one is that scoring requires a lot of time and energy with a large number of papers and a time limit for completion, and the other is that the objectivity of the scoring may not be guaranteed. When a large number of translated answers are needed to be evaluated, the grading criteria may change with the subjective feelings of teachers. As a result, it is necessary to implement automatic scoring of translation results submitted by students. Therefore, there is a need for automatic scoring of translation results submitted by students. Automatic scoring for translations can greatly improve the efficiency of students' translations results scoring, reduce the tedious work of manual scoring, and lower the impact of teachers' personal subjective feelings on the scoring results through using automatic metrics.

Automatic evaluation is generally based on objective evaluation metrics, which can be analogous to automatic evaluation in machine translation. According to the research results in [1], BLEU [2] is used in 98.8% of machine translation evaluation papers, and it is mainly calculated by the similarity between students' translations and reference translations. There are similarities between machine translation and dialogue systems, that is, the source language statements of machine translation correspond to the query of dialogue systems, and the target language statements correspond to the reply [3]. As a consequence, some evaluation metrics of machine translation are often used in the evaluation of dialogue systems although they are later proved to be less relevant to human judgments [4]. Inspired by the idea, this paper tries to apply automatic evaluation metrics in dialogue systems to translation scoring for English education, aiming to reduce efforts of correcting translations by hand.

Inspired by Deep AM-FM [3], a good translation should fully translate the semantic content contained in the original sentence and keep fluent. Therefore, this paper evaluates the quality of translations from the perspectives of accuracy and fluency. The contributions of this paper are mainly as follows:

1. The translations scoring is linked with dialogue systems, and the evaluation metrics of dialogue systems are applied to automatic scoring for translations. Two appropriate dialogue evaluation metrics, RUBER [5] and HolisticEval [6], are selected to score the accuracy and fluency of students' translations, respectively, and slight changes are made according to [7].
2. Several heuristics are used to combine the accuracy and fluency scores by the two metrics. Additionally, the hybrid metric is applied to automatic scoring of translations, and then we analysis the correlation between hybrid scores and human judgments on a collected dataset.
3. We conduct a case study in which a representative selection of submitted translations from the collected dataset visually demonstrated the differences between the four which are accuracy scores, fluency scores, hybrid scores, and human scores.

The structure of this paper is as follows: Section 2 mainly discusses the related work, which consists of two parts: automatic scoring for translations and evaluation metrics for dialogue systems; Section 3 introduces the method and processing steps of two metrics which are used. Then, Section 4 presents the results of experiment, including a case study on automatic evaluation of students' translation results with the hybrid metric; additionally, the threats and future directions of our research are discussed in Section 5 and the conclusion is drawn in Section 6.

## 2. Related Work

We focus on the work related to automatic translation scoring for English education. And the research is mainly carried out from two aspects: automatic translation scoring and evaluation metrics of dialogue systems.

### 2.1. Automatic Scoring for Translations

There are two main types of automatic scoring methods for translations: scoring translations using certain models, or scoring translations by cross-referencing with references. The former does not require cross-referencing with a reference translation but only a trained translation scoring model, while the latter does not require a trained model but a reference translation. Compared with manual scoring, the automatic scoring method has the advantages of speed and efficiency, but the scoring results often do not fully reflect the quality of the translation and still have shortcomings.

Guzmán et al. [8] proposed a neural network-based evaluation method, which can select the best translation from two candidate translations to be evaluated based on the reference translation. This evaluation method can integrate the syntactic and semantic information of the reference translation and the characteristics of the two candidate translations to find out the translations with higher translation quality from the candidate translations, but it cannot give a specific score.

Gupta et al. [9] proposed a machine translation evaluation method based on dense vector spaces and recurrent neural networks (RNNs), which can give specific evaluation scores to the translations to be evaluated. The method obtains dense vector representations of the reference and translation through recurrent neural networks and predicts the similarity scores of the two based on a neural network which considers both distance and angle between the reference and translation.

Tian [10] has designed an English-Chinese translation system for students online automatic grading and providing intelligent feedback, including automatic grading module rating from vocabulary and sentence patterns. The former uses different methods according to the part of speech of the words, consisting of synonyms matching and similarity calculation, and the latter compares with the sentence patterns of reference translations. The final score is a blending of the words and sentence patterns with their respective scores.

Unlike [10], Zhang et al. [11] do not use a reference translation. They proposed a multitask learning QE model to score and rank translations. In the scoring task, the model calculates the cosine similarity between the source language sentences embedding and the target language sentences embedding as the translation score instead.

Designing effective features plays a key role in automatic scoring for translations. Shah et al. [12] proposed some translation features obtained through neural network training, which can be used for translation quality assessment, including continuous space language model features, word vector features obtained from large-scale monolingual corpus training, and similarity score features between target language words and their pairs of source language words obtained by word alignment calculation. These features are trained by unsupervised methods, which are simple, efficient, and highly adaptable.

In the process of research, we found that (1) there is relatively a few work about automatic scoring for English education; (2) most of them rely on comprehensive systems without focusing on evaluation metrics; and (3) the research is not in-depth enough, and relevant papers do not have high qualities.

### 2.2. Metrics of Dialogue Systems

Metrics are usually used to evaluate the quality of the response generated corresponding to a given query in dialogue systems. They can be divided into the referenced and unreferenced according to whether ground-truths are needed, which is similar to whether reference translations are needed in automatic translation scoring. As a consequence, the metrics of dialogue systems can be used to automatically grade students' translation results.

#### 2.2.1. Referenced Metrics

ADEM [13] used a hierarchical RNN encoder to encode the context, model response, and reference response and used the square of the difference between human scores and model scores to constantly adjust parameters. However, this method needs a lot of human annotations, which is really time-consuming, and the predicted scores of the model are generally low.

Deep-FM [3] measures the quality of responses from adequacy and fluency: ① take the maximum cosine similarity between model responses and different reference responses as the adequacy score; ② take the ratio of the minimum and maximum probability of model responses and reference response as the fluency score. The whole idea of this method can provide some inspiration for our research.

Similarly, Lan et al. [14] analyzed the existing dialogue evaluation methods from three aspects of fluency, coherence, and engagement. Moreover, they proposed a new method that can solve the drawbacks of negative sampling, which also makes use of the ground-truth.

#### 2.2.2. Unreferenced Metrics

Both of metrics mentioned above require reference responses, but GRADE [15] does not. It gains contextualized representations in the utterance-level and dialogue graph representations in the topic-level. However, what we expected is to evaluate the quality of translation sentence rather than the topic transition dynamics.

Pang et al. [6] proposed comprehensive dialogue evaluation metrics from four aspects of context coherence, fluency, diversity, and logical self-consistency, respectively. The evaluation method of dialogue fluency here is similar to Deep AM-FM [3], while the language model used is better and consequently can provide the foundation for our work. Considering the attributes that need to be evaluated in translation scoring, we choose the fluency and accuracy of translations as the characteristics of scoring students' translation results.

## 3. Method

In order to achieve automatic scoring for students' translation results, this paper used a combined objective metric, which is a hybrid of accuracy score and fluency score of a translation. Several heuristic methods are intended to mix the automatic scores of the two metrics and the correlation with the human scores will be used as a measure of these methods. The final hybrid score consists of two parts in the overall framework, translation accuracy and translation fluency, which are automatically scored by selected metrics. The overall framework of the methods is shown in Figure 1.

### 3.1. Translations Accuracy

Teachers usually assign scores to the translation results based on the referenced translations and their experience in the actual process of translations scoring. This section makes use of an automatic evaluation metric to reduce human efforts according to reference translations. And the similarities between the translation results submitted by students and the referenced translations are the key point of scoring, which is defined as the accuracy of the translation in this paper. Consequently, we need to select the language model with excellent performance to generate word embeddings of sentences in preparation for computing the similarities between them. The main disadvantage of Word2vec is that it only provides static vector of words; that is, it can only generate fixed vector representations for words with multiple semantics [7].

However, the pretrained language model BERT [16] can solve the polysemy problem of a word. BERT [16] is composed of Transformer encoders, which can realize bidirectional encoding in real. The corresponding unsupervised training tasks masked language model (MLM) can realize bidirectional context representations, which differs from that of the separate left-to-right and right-to-left language models [16]. The MLM randomly blocks a certain percentage of the input tokens and then predicts the masked tokens on the basis of unmasked context tokens, so that the representation takes into account both the left and right context [16]. This paper mainly uses BERT [16] to generate contextualized word vectors.

Algorithm 1 presents the approach to obtain the accuracy scores of students' translations. Firstly, the word vector representations of sentences are needed to obtain. According to the analysis of [7], the model BERT [16] is more competitive than any other; therefore, it is chosen to replace Word2vec in [5] to generate the word embeddings of sentences. Secondly, the elements of each vector will be taken the maximum and minimum values in terms of the column to form new vectors, which are pooling strategies that can summarize and simplify information. Then, the new vectors are supposed to be concatenate in order to obtain new representations of the sentence. Both students' translations and reference translations need to go through the same processes. Finally, the cosine similarity of the two sentence vectors is taken as the accuracy score of student's translation, which means that the larger the value is, the more similar two sentences are. And the equation of the cosine similarity [5] is as follows:

(1) $$\begin{array}{c} \text{cos}\left(v_{s},v_{r}\right)=\frac{v_{s}^{T}\;v_{r}}{\left\|v_{s}\right\|\cdot \left\|v_{r}\right\|}, \end{array}$$

where *v*_*s*_ is the new vector of student's translations after pooling, and *v*_*r*_ is the new vector of the corresponding referenced translation.

### 3.2. Translations Fluency

In addition to translation accuracy, fluency ought to be ensured for a good translation. Xu et al. [17] believe that fluency represents the possibility of text being generated by human beings in the research of text generation, which is also applicable to our work about evaluation of translations. Stumbling sentences will affect the score of a translation. According to [6], the negative perplexity of translation results is taken as fluency scores. In essence, it is negatively correlated with the probability of sentence. The calculations of fluency do not need the referenced translation as an auxiliary but only calculate the corresponding fluency of translations which are submitted by students, mainly to investigate whether sentences are smooth and correct grammatically.

In order to calculate the fluency scores of translations, we will calculate the probability value of the sentence to be tested through the pretrained language model after inputting the sentence to be tested and then normalize the result to make the value range from 0 to 1 between. In this paper, we choose Pretrained Transformer 2 (GPT2) [18] as the pretrained language model. GPT2 [18] is a large Transformer-based model [19] that can generate coherent text passages and can accomplish many different language modeling tasks such as reading comprehension, question answering, and machine translation without pretraining. The GPT2 [18] model consists of the decoder part of the multilayer unidirectional Transformer and only uses multiple masked self-attention and feed forward neural network modules. It predicts the next word through the input sentence and then adds the new word as a new input to continue the prediction. The loss function calculates the deviation between the predicted value and the actual value.

Algorithm 2 shows the approach to obtain the fluency scores of students' translations. Drawing on the experience of previous studies, we calculate probability values through GPT2 [18], which is an excellent pretrained language model. Nonetheless, the model has not been fine-tuned, which is a slight difference from [6]. Firstly, the required model and vocabulary are loaded and initialized by calling relevant classes of the pretraining model. In this step, we import the packaged GPT2LMHeadModel and GPT2Tokenizer in the pytorch_pretrained_bert library as the pretrained GPT2 model. Secondly, students' translations need to be encoded and converted into forms. For the sentence to be tested, use GPT2Tokenizer to create a tokenizer object, encode the original sentence, and convert it into a tensor. Then, the tensor obtained after encoding the sentence to be tested is passed into the GPT model, and then the results will be input into our model in order to obtain the initial fluency scores. And the initial fluency scores [6] are gained by

(2) $$\begin{array}{c} f\_\text{initial}=\frac{1}{n}\sum_{t}^{n}\text{log}P\left(s_{t}|s_{\langle t}\right), \end{array}$$

where *n* is the number of tokens in student's translation, *s*_*t*_ is the *t*_*th*_ token of student's translation, and the *P* denotes the model GPT2 [6].

At last, we normalize the resulting fluency scores. Different evaluation metrics often have different dimensional units, and this will affect the results of data analysis. In order to eliminate the dimensional influence between different metrics, data normalization is required to solve the comparability problem between measures. After the original data are standardized, the metrics are in the same order of magnitude, which is suitable for comprehensive comparison and evaluation. We normalize the scores to values in the range of 0-1 by using a formula in [6], which defines the lower bound as the fifth percentile.

## 4. Experiments and Results

### 4.1. Datasets

We selected 10 moderately difficult middle school Chinese-English translation questions from baiduwenku (these questions and references are come from https://wenku.baidu.com) and corresponding referenced translations. They contain a variety of sentence patterns, such as declarative sentences, interrogative sentences, and exclamatory sentences. Then, we obtained English translations after showing just Chinese to ten volunteers. Then, we obtained English translations after showing just Chinese to ten volunteers. As a result, there are 100 translations in our dataset, including four empty sentences, which are not eliminated in that this is what might happen in translation problems.

### 4.2. Human Scores

Two graduates were invited to score for volunteers' translations by combining their English knowledge with references. They were demanded to rate translations from the accuracy and fluency and give a total score of every translation. And they need to combine their own knowledge and the referenced translations to score the translation results submitted by students of the dataset on a scale of 0–5 (from very poor to very good). As a consequence, human scores are the average of two people's scores. Afterwards the Min-Max normalization is used for mapping the resulting values to [0, 1].

### 4.3. Steps

After the preparation of our dataset and human scores, we plan to reproduce the two metrics so as to obtain objective scores of students' translations. We chose Python for the language support because of its power of functions and the simplicity of syntax. The detailed implementation steps are as follows.

#### 4.3.1. Accuracy

1. Download and install required software and packages for Windows.
2. Locally download the pretraining language model released by Google, and then start the BERT service on the server.
3. Use the language model BERT to encode sentences in the dataset to get vector representations.
4. Make the max-pooling and min-pooling.
5. Program the function of the cosine similarity in order to obtain the score of the translation. When one of the two sentences is empty, the similarity score is directly set to 0.

#### 4.3.2. Fluency

1. Import the pretrained GPT2 model.
2. For the sentence to be tested, it is firstly segmented, and based on the result of the segmentation, the original sentence is encoded and converted into a tensor.
3. The tensor obtained after encoding is passed into the GPT2 model, and the fluency score of the sentence is calculated. If the sentence to be tested is empty, then it will be set a score to 10^6^ (normalize the score).
4. The score is normalized to be in the range of 0-1. It should be noted that the fluency scores obtained directly may be negative, and the distribution of scores varies from dataset to dataset, which is normalized according to the formula defined in [6].

### 4.4. Results

In order to demonstrate the feasibility of using the two metrics of dialogue systems for scoring translations, we draw several scatter plots to observe the correlation between scores based on metrics and human. What calls for special attention is that we randomly added a perturbation of 0.05 to human scores to make it easier to observe the effect due to repetitive scores. Moreover, we discard the points where the score is 0. As shown in these figures, we find the following:

- Figure 2 shows the scatter plots between metrics in [5–7] and human judgments in terms of accuracy and fluency. From both sides, the scores of metrics are correlated with manual scores. However, it can be seen that accuracy scores are higher than human judgments on the whole, which are generally above 0.9, while fluency scores are much lower than human scores with the highest score not exceeding 0.7.
- The difference is that Figure 3 is for two metrics and human scores in total. A similar conclusion can be drawn from Figure 3, which the two metrics are not suitable to be used as the scoring standard for translations alone.
- Besides, Figure 4 shows scores between humans and mixed by two metrics in several ways. The figures show the arithmetic average, geometric average, or a mixture of different proportions of two scores. It can be seen that scores are closer to human scores after mixing. There is a little difference on the effect between arithmetic mean and geometric mean; however, the former is susceptible to the influence of extreme data.

### 4.5. Case Study

Considering the correlation between translation scores and response scores generated by dialogue systems, we refer to the metrics related to the evaluation of dialogue systems. To give a clearer picture of the feasibility of this inspiration, we selected five examples and gave their accuracy, fluency, and human scores. At the same time, we used different methods to hybrid the two parts of scores to select which is the most similar to human scores.

As is shown in Table 1, we can draw the following conclusions: (1) the accuracy scores are generally high, and scores of different quality don not differ much. The reason may be that the method of calculating accuracy scores is based on the embeddings, which sentence representations are fuzzy [14]. In addition, we take the average of all accuracy scores in our dataset, and the result is 0.90082, which includes four empty sentences whose scores are 0. As a consequence, it can be concluded that the embedding-based metric is not suitable for scoring translations alone. (2) The fluency scores are generally low on the contrary, but it is basically consistent with human scores, which can replace them in terms of fluency to some extent. The average of fluency scores is 0.27875, which is also not suitable for the total scores of translations alone. (3) According to the results of mixing the two fractions in Section 4.2 in several ways, we directly select the geometric mean of scores to display here. It can be seen from the table that the hybrid scores have a great correlation with the human scores.

## 5. Discussion

The conclusions obtained from scatter plots and the case study can be verified by each other. The scoring rules of the two metrics we selected are roughly the same as human scoring in terms of accuracy and fluency of translations; however, the former is on the high side while the latter is on the low side. The two metrics are not suitable for translations scoring independently, but their hybrid scores are closer to human judgments.

We summarize the internal and external effectiveness threats of this method as follows.

Threats to external validity are related to the quality of the datasets we collect. Our experimental data come from the English translation results of ten Chinese sentences collected from ten volunteers, a total of 100 translations. More experimental data can better prove the universality of the experimental results. In the future work, we can collect more translations and provide a larger translation dataset. Besides, in addition to the translation from Chinese to English, it can also be extended to other languages.

Threats to internal validity include the effectiveness of selected dialogue evaluation metrics and the impact of heuristic methods of mixed measurement on scoring quality. Firstly, in this paper, we choose two metrics in the field of dialogue system, including the accuracy metric proposed by RUBER [5] and the fluency metric proposed by HolisticEval [6], to evaluate the quality of translations. Both of them are based on embedded metrics. However, according to the experimental results of [14], the metrics based on learning is better than the metrics based on embedding. Therefore, we will consider applying better dialogue evaluation metrics to automatic scoring to improve the efficiency of translation scoring. In addition, we also use some heuristic methods to mix the two metrics, but the difference in effect is not particularly obvious. Therefore, in future work, we will learn the weight of each score through the model and optimize the mixed results of the two metrics. We look forward to developing our own translation scoring standards to reduce the workload of future English teachers.

## 6. Conclusion

Since there are some similarities between the quality assessment of responses generated by dialogue systems and the quality evaluation of translations, we are inspired of using the automatic metric of dialogue evaluation to measure the quality of translations in English education, in order to reduce the time and efforts spent in manual scoring and improve the objectivity of the scoring. In this paper, we select the referenced metric in RUBER [5] and the fluency metric in HolisticEval [6], refer to [7] to make some improvements on the original basis, and then apply them to the translation scoring. The experiments prove that the mixed results of the two are applicable to the scoring process of students' translation results, and translation scoring automation can be realized depending on the system. It can reduce the efforts of manual scoring and improve the efficiency and fairness of scoring.

## Figures and Tables

**Figure 1:** The overall framework of the methods.

**Figure 2:** (a) Correlation of scores by the metric with the human rating in accuracy; (b) correlation of scores by the metric with the human rating in fluency.

**Figure 3:** (a) Correlation of accuracy scores by the metric with the human rating in total; (b) correlation of fluency scores by the metric with the human rating in total.

**Figure 4:** (a) Correlation of the arithmetic mean of two scores by the metric with the human rating in total; (b) correlation of the geometric mean of two scores by the metric with the human rating in total; (c)–(h) correlations of the accuracy and fluency scores on a 2/8, 3/7, 4/6, 6/4, 7/3, and 8/2 ratio mixed with the human rating in total.

**Algorithm 1:** The approach of obtaining accuracy scores for students' translations.

**Algorithm 2:** The approach of obtaining fluency scores for students' translations.

**Table 1:** Translations submitted by volunteers from our dataset. Hybrid scores are the geomean of accuracy scores and fluency scores.

Questions	Translations	References	Accuracy	Fluency	Hybrid	Human
七十周年阅兵式壮观的景象将永远铭刻在我的脑海里	I will be remember the scene about the 70 year's	The grand sight of the 70 anniversary military parade will be forever impressed on my mind	0.893304	0.074850	0.258580	0.3
店主在卖这台空气净化器时向你开价多少?	What is the price of the xx sold by the seller?	How much did the shop owner charge you for the air cleaner?	0.905867	0.232175	0.458606	0.4
不要运动过度，不然有猝死的可能	If xxx, you may die at once	Don't exercise too much, or you may die of sudden death	0.864336	0.101226	0.295793	0.4
如果有朝一日学生能亲自参与到课程开发中, 那该有多棒啊!	How wonderful it would be if one day students could personally participate in the course development!	How great it is if one day students can be involved in the development of courses on their own!	0.955349	0.398698	0.617167	1.0
生态保护对人类的福祈和未来至关重要, 也孕育着世界发展的历史性机遇	Ecological protection is crucial to the well-being and future of mankind. It also breeds a historic opportunity for world development	Ecological protection is essential to human beings well-being and future, which also brings about the historical opportunity of the world's development	0.958789	0.380757	0.604206	0.8

## Data Availability

The data used to support the findings of this study are available from the corresponding author upon request and at https://github.com/ghj9922/Automatic-scoring-for-translations-based-on-language-models/tree/main.
